# Prediction Model of Rice Seedling Growth and Rhizosphere Fertility Based on the Improved Elman Neural Network

This article has been retracted.

**DOI:** 10.1155/2022/2151682

**Published:** 2022-07-31

**Authors:** Feng Jiao, Yang Chen, Xinyue Zhang, Yuyue Zhou, Linlin Wang, Jinhua Wu

**Affiliations:** Heilongjiang Bayi Agricultural University, Daqing, Heilongjiang 163319, China

## Abstract

Rice developing prognostication is a key part of precise agricultural management, and its advancement is an intricate course of events involving the interplay of breed and environmental element. The traditional research method is based on data analysis of rice growth prediction modeling, mining the concealed rapport between rice productivity and circumstance element, for instance, weather, sunlight, and water, and then predicting its yield and analyzing the complex rapport between the circumstance element and growth in every developing phase. In this dissertation, the improved ElmanNN is accustomed to establish a prediction model, and the ElmanNN is accustomed to determine the rapport between the circumstance element and growth in every developing phase simultaneously so as to avoid the arithmetic falling into local optimum easily. In this dissertation, the improved genetic arithmetic is accustomed to optimize the initial weight and threshold of Elman neural network, and the range of weight value multitudinous layers in the mould are obtained by training the network with samples that have been tested in the last few years. Finally, the rapport between growth and yield in six different periods is independently modeled, and the training samples are build up separately one by one based on physiological parameters and environmental indicators of rice at every level. The experiments show that the accuracy for the prediction model in the light of the improved ElmanNN has been beneficial.

## 1. Introduction

Since ancient times, rice has been one of the most important “rations” in my country, and the people's food has always been closely related to social stability [1]. With the acceleration of urbanization, the area of cultivated land continues to decrease. It is particularly important to use limited land resources to produce more high-quality rice. It is not only related to social stability but also directly related to national food security [2]. Compared with many crops, rice has a long growth process, relatively large part growth cycles, complicated high-yield management points, great changes in morphological and physiological characteristics in different cycles, and many factors affecting growth. For a long time, people's judgment on the growth situation of rice is mostly based on experience summary [3]. Therefore, accurate prediction of rice growth and development has important practical significance, and it is also an important research front of precision agriculture and modern agriculture.

These days, with the high-speed upgrowth of info technology, especially the development of Internet of Things technology, embedded technology [4, 5], ZigBee technology, cloud computing, and other technologies [6], Internet technology has become more and more important in agricultural production. The application has become a reality, and “Internet + rice” has become a new model to promote agricultural production and farmers' income. At present, the paddy field management systems on the market still rely on manual control. They often require users to preset one or more ranges of plant growth indicators based on experience values, and then the system will adjust each growth parameter according to the preset values to maintain the growth of the plants within the growth range [7]. In the actual use, experienced farmers will continue to manually adjust the parameters to meet the environmental requirements of multitudinous growth stages of rice, such as the water level does not overflow the top of the plant during the greening period, and the shallow water layer is accustomed to wash the fields during the grain-filling period. However, no matter how timely the manual adjustment is, there is still a certain lag, so it is not realistic to rely on the preset index value of manual experience value to achieve high rice productivity. Therefore, a practical and efficient rice developing prognostication system is urgently needed to help users understand the growth situation of rice in this environment in advance and even to estimate the final yield of the season, providing users targeted regulation of circumstance element on a scientific basis.

In summary, based on the preceding discussion on the collision of circumstance element on rice development, this thesis focuses on analyzing the progress characteristics of paddy in multitudinous development phases and gives a definition of paddy developing that takes into account the expansion period and key developing indicators of each stage. Paddy developing is an overall indicator that uses a numeric value to characterize the growth outcome within a given time spacing. The paper uses the neural network modus to study the rapport between various circumstance elements and paddy developing and uses the growth value to represent the growth, which lends a up to date cogitation for the prediction of paddy developing. The rice developing prognostication model established in this dissertation has a certain research value and social value.

## 2. Research Status at Home and Abroad in the Field of Rice Growth Prediction

In the light of the analysis of great amount of rice growth test data, it is found that a relatively large part of related factors affecting rice growth are interrelated and affect each other. The rapport between the growth potentials of different periods is entangled with each other, which cannot be explained by one or two mathematical formulas. It is a multifactor and nonlinear problem. Statistical models and crop growth models are the most common and effective methods in agriculture to assess the collision of circumstance element on agricultural production [8, 9]. The predecessors have carried out many discussions on the rapport between weather changes and crop yields, but they mostly focussed on the simulation and prediction of crop yields under changing scenarios based on meteorological factors such as temperature and precipitation. The research modus are mainly linear statistical simulation methods and climate models. Numerical simulation modus nested with the crop model [10–12]. Most of the studies on soil moisture on rice productivity are still at the stage of relying on empirical models, conceptual models, and mechanistic models [13]. Yin used the winter wheat yield in Weinan City and meteorological data over the years as data sources, further decomposed and calculated the actual yield [14], and quantified meteorological factors such as precipitation, light, and accumulated temperature in multitudinous developing phases by using the linear weight of the sample from the forecast year. Finally, the output prediction model was synthesized through the regression equation, and the simulation results were compared with the measured output, and the two were in good agreement. Zhang studied the data of rice plant traits at multitudinous growth stages in 11 sowing dates in Shanghai, and combined with the theory of accumulated temperature [15], he measured the effective accumulated temperature of multiple growth stages and established the dynamics of paddy developing traits on this basis. The model can further simulate the dynamic changes of rice stems and tillers, leaf age and grain filling, and has a good simulation effect. Cheng integrated the data and environmental data such as temperature, humidity, and illumination inside the greenhouse and local weather conditions [16] and established a global variable prediction model for the future environmental conditions of the greenhouse through the neural network modus, which solved the problem in the conventional greenhouse control scheme. Due to the relatively independent working places, the setting adjustment of each actuator is delayed. The experimental comparison results show that the greenhouse intelligent control system based on this model is more reasonable and stable. Aiping selected wheat yield data in dry farming areas in my country as a sample, combined with BP, RBF, and GRNN neural network models, and used the IOWA operator to propose a combined neural network model for predicting wheat yield [17, 18]. After comparing the prediction models, it is found that the combined model has higher accuracy and the best prediction effect. Mechanism-based methods for predicting paddy developing require a large amount of very detailed data and knowledge from multiple agricultural disciplines and are difficult to achieve. Through the analysis of the current situation of rice developing prognostication at home and abroad, this paper chooses to use the neural network to conduct research on rice developing prognostication.

Rice developing prognostication helps to quantitatively assess the growth potential of paddy. The established rice developing prognostication model is helpful for analyzing the rapport between paddy developing and circumstance element and provides a basis for adjusting various growth factors like weather, light, heat, and fertilizer to improve rice productivity. With favorable support, users can understand the current development status of rice based on the predicted results, especially whether the rice is healthy. After studying a number of existing literatures on the growth features of paddy in multitudinous development phases, and considering the difficulty of realizing the project, it was decided to use the neural network as a powerful tool to study the comprehensive influence of circumstance element on paddy developing. At present, BP neural network, as a relatively mature artificial intelligence arithmetic has a good nonlinear mapping ability and generalization ability and is widely used by scholars in prediction of paddy developing and yield, but the evolution prediction of rice belongs to time. For the sequence prediction problem, ElmanNN has better state transfer ability, so ElmanNN is a better choice than the BP neural network.

## 3. Rice Growth Prediction Model

The paddy developing model in a broad sense is a dynamic mathematical model that integrates factors such as soil, variety, climate, and cultivation methods [19, 20]. The research on the paddy developing prediction model in the paper focuses on the prediction of the influence of various circumstance element such like weather, rainwater, degree of heat, and nitrogen content on the upgrowth of paddy in multitudinous development phases and evaluates the growth conditions of different stages to obtain the final rice productivity of this season. The research method used in this dissertation is a neural net, so a large number of samples are in demand to train the model, and the weights are constantly adjusted, and finally, the rice growth prognosis model is acquired. The process of establishing and using the model is shown Figure 1.

### 3.1. Circumstance Element of Rice Growth in Different Growth Stages

#### 3.1.1. Effect of Temperature on Growth

Each developing phase of rice has its own temperature requirements. If the temperature rises above the biological maximum temperature of each developing phase, it will have a negative effect on the normal growth and development of rice and even causes “heat damage.” High temperature at the jointing and booting stage of rice mainly affects the development of flower organs, affects the differentiation and degradation of spikelets, shortens the length of spikelets, and inhibits enrichment, resulting in a decrease in grain length and grain width and a serious decline in the weight and quality of rice grains. If the temperature drops below the minimum temperature of each developing phase, the phenomenon of “chilling injury” will also occur. When rice is subjected to low temperature stress, especially during the flowering period, the tapetum will become thicker and nutrient imbalance will cause pollen to lose fertility, affecting pollen vigor, quantity, and the process of spikelet pollination and fertilization, resulting in poor flowering and pollination of rice, grain abortion, and grain filling. When obstructed, empty, half-empty, and black particles increase, the output drops sharply.

#### 3.1.2. The Effect of Moisture on Growth

Rice has different degrees of water sensitivity in different growth stages. Studies have shown that the greening stage, jointing booting stage, and heading and flowering stage are relatively sensitive to the water response. The heading and flowering stage is the most critical period for rice growth. At this time, the physiological water demand is more sensitive. The lack of water at this time may cause the pollen to die during pollination, affect pollination to form empty shells, and easily cause premature aging of roots and leaves. The grain-filling period is the peak of vegetative growth of rice. The lack of water at this time will directly weaken the photosynthetic efficiency of leaves and affect the production of plant organic matter and nutrient transport, resulting in insufficient grain-filling and reduced grain weight. However, if the irrigation is too deep, the roots will be flooded for a long time, which will affect the vitality of the roots, resulting in hypoxia and premature nutrient aging of the plants.

#### 3.1.3. The Effect of Light on Growth

Light is an important meteorological factor for rice productivity and quality. Light intensity has a very significant collision on the photosynthetic rate, transpiration rate, and saturation point of plants. Especially the sunshine hours during the flowering and grain-filling stages have a significant effect on the yield and quality of rice which is closely related [21]. Generally speaking, under the condition of constant temperature, high light conditions are beneficial to increase the photosynthetic rate of rice plants and promote growth and development, and sufficient temperature and light are beneficial to the growth of rice seedlings and promote early tillering and rapid development, while low light adversity reduces the rate of plant growth. The net photosynthetic rate leads to a slowdown in the production and accumulation of dry matter, and the plants are greedy and late, resulting in a decrease in the final yield.

### 3.2. Construction of an Improved Elman Rice Growth Prediction Model

ElmanNN by Jeffrey L in 1990 [22, 23] because of its excellent performance has a lenient scope of submissions in medium and long-term weather forecasting, power grid load optimization, object recognition, and other application models that have high requirements for computing power and accuracy. It usually consists of four layers: input layer, hidden layer, receiving layer, and output layer. The input layer sporting the part of signal transmission; the output layer sporting the part of linear signal weighting; the hidden layer sporting the part of abstraction, abstracting and extracting input features for better linear division of different types of data; the succession layer sporting the part of delay operator memory. The hidden layer outputs the value just before and is self-connected to the input of the hidden layer. This internal give back method heightens the capability of the network itself to process dynamic info, and the effect of moving model is good. The specific fabric of the neural network is shown in Figure 2.

The mathematical characterization of the ElmanNN is abided by formulas (1)–(3), where *x*(*k*) is the output of the hide layer, *X*_*c*_(*k*) is the manufacture of the neuron node in the middle layer, *y*(*k*) is the network output, and *α* is the self give back gain factor. *f* is the transfer function of neurons in the hide layer. The common transfer function is the *sigmoid* function. *W*^1^, *W*^2^, and *W*^3^ are the degree of seriousness between the input layer and the hide layer, the successor layer to the hide layer, and the hide layer to the output layer, respectively. Vector, *g*, is the linearly weighted transfer intention of the output neuron.

(1) $$\begin{array}{c} x_{c}\left(k\right)=\alpha x_{c}\left(k-1\right)+x\left(k-1\right), \end{array}$$

(2) $$\begin{array}{c} x\left(k\right)=f\left(W^{1}x_{c}\left(k\right)+W^{2}\left(u\left(k-1\right)\right.\right), \end{array}$$

(3) $$\begin{array}{c} y\left(k\right)=g\left(W^{3}x\left(k\right)\right). \end{array}$$

Compared with the most commonly used BP neural network model, ElmanNN has the ability of dynamic feedback, which not only heightens the capability of the network to map the transfer function but also improves the convergence accuracy of the network. It can already initially meet the normal use requirements. However, in the experiment, it was found that there are very few points and the expected results are far from the expected results, the trend of change is opposite, and this phenomenon does not occur every time. After careful analysis of the reasons, we believe that at some point, the ElmanNN may be trapped in local extrema. After careful study of the defects of ElmanNN, it is found that the primary weights and thresholds of the net are generatic by stochastic arithmetics, such as the Nguven–Widrow arithmetic because it has no reasonable initial parameters for network training in the field of paddy developing prediction. In addition, the ElmanNN in the paddy developing prediction model here uses a gradient descent learning arithmetic. Once the initial given range is not good, the network is happy to land oneself somewhere a local optimal solution. Therefore, the direction of the next majorization is very clear. By changing the stochastic of the initial repetition and thresholds, the accuracy of the prediction model can be further improved.

## 4. Based on the Improved ElmanNN and Its Application in Rice Prediction

Since the initial weights and thresholds of the standard ElmanNN are randomly generated, when the gradient descent arithmetic is used as its learning arithmetic, the arithmetic is easy to fall into the local optimal solution. On this basis, this paper proposes a genetic arithmetic and ElmanNN fusion arithmetic. The genetic arithmetic is accustomed to select and optimize the initial network parameters of the Elman network in the rice growth prediction model. The probability is corrected to further improve the performance of the arithmetic.

### 4.1. Improved Genetic Algorithm to Optimize ElmanNN

The training and learning method used by ElmanNN is usually the gradient descent arithmetic, which requires that the error function must be continuously differentiable so that the solution of the problem moves from the current position in the search space to another position along the negative direction of the error gradient, and the search direction is relatively low. This makes the performance of the network mainly depend on the selection of the initial weights and values [24]. However, the initial values are randomly selected. In complex or multiextremal data, improper selection will cause the neural network to fall into the local optimum state. Aiming at the defect of poor global search ability caused by the ElmanNN gradient descent arithmetic as the benchmark in the rice growth prediction model, it is easy to fall into local extreme points, the paper introduces the genetic arithmetic to train and correct the weights and thresholds of the Elman network, which can be used in complex. In the large amount of rice environmental data, the global optimal solution of the problem is searched with high efficiency, which greatly reduces the possibility of falling into the local minimum value.

### 4.2. Comparative Analysis of the Prediction Effect of Rice Growth

The experimental data in this dissertation are processed by exception processing and normalization before being input into the model so as to illustrate the effectiveness of the ameliorate. ElmanNN in the paddy upgrowth prediction mould, and a set of sample data in the greening period of the test set was taken as an example. The data were input into the model after exception processing and normalization processing. Model prediction accustomed BP neural net, criterion ElmanNN, and ameliorate ElmanNN. In this experiment, the input is the environmental index and the number of days of growth, and the output is the growth amount at this stage. To study the collision of different environments and management methods on the growth of rice in the greening period, we can first approximate the physiological indicators of the rice in the greening period. The weight coefficient *F* of the influence of rice growth during the period is 14.41%, 10.56%, 12.27%, 35.03%, and 27.3%, and the rice can be obtained by multiplying the weight coefficient F by the corresponding physiological evaluation index value. When the ameliorate genetic arithmetic optimizes the initial weights and sills of ElmanNN, the initial parameters have a bigger effect on the optimization outcomes. Here, the initial colonial dimension of the genetic arithmetic is set to *M* = 100, the maximum genetic algebra = 200, and the overlapping odds and sudden change probability are automatically regulated by the adaptive arithmetic in the previous section.

It can be seen from Table 1 that the astringent accurateness of the net when the calculation of nodes in the hide layer is 7 in the greenback period model is first-rate. Therefore, the calculation of selected point of intersection is 9. The same way, this method is also accustomed to calculate the five-upgrowth-stage mould such as tillering phase, and it is found that the best result is 9. Therefore, the calculation of hide layer nodes of the five-upgrowth-phase models such as tillering level is 9, and the hidden layer of the overall model is 9. The calculation of nodes is 7. In this dissertation, relative failing, MSE, and MAE are accustomed to compare and analyze the accuracy of inherited BP neural net, criterion ElmanNN, and ameliorate ElmanNN in the process of rice growth prediction. Simulation errors of three kinds of neural are compared. Relative error, MSE, and MAE are accustomed to compare and analyze the accuracy of inherited BP neural net, criterion ElmanNN, and ameliorate ElmanNN in the process of rice growth prediction. Simulation errors of three kinds of networks are compared, and the results are shown in Table 2.

Due to the perspective of mistake analysis, as shown in the table, compared with the inherited BP and ElmanNN, the ameliorate arithmetic has a tiny error scope, and simultaneously, the points with larger prediction errors are smaller and the volatility is smaller, which extremely improves the prognostication accuracy. By the perspective of astringent speed, as shown in Figure 2, the ameliorate arithmetic gradually stabilized 150 steps, while the Elman neural network took about 250 steps to accomplish the convergency. It can be seen that in the ameliorate ElmanNN, the convergence rate is faster than that of Elman. Therefore, the prediction effect of the ameliorate ElmanNN in the rice growth prediction model is better than that of the standard ElmanNN and the inherited BP neural network. The prediction outcome of the three neural networks is as follows. The prediction value of the inherited BP neural has a low degree of fit with the change in trend of the actual data, and some fallacious points exist. The prediction value of the criterion ElmanNN has a good arithmetic accuracy. However, there are still individual error points with the opposite trend, indicating that the ElmanNN will still be trapped in local extreme points, and the Elman's fitting degree has been ameliorated by the genetic arithmetic.

## 5. Conclusion and Outlook

The growth of rice is a relatively intricate dynamic handle, which is affected by various circumstance elements such as light, weather, and rainwater so as to achieve the purpose of accurately predicting the upgrowth of rice in each developing phase, and this thesis proposes a rice growth model based on improved ElmanNN, and it applies this method to rice growth prediction.

### 5.1. Summary

1. The paper defines the concept of rice growth for the first time to quantitatively describe the growth of multitudinous growth stages. This paper introduces the significance of rice growth prediction and the current research status at home and abroad in the field of rice prediction, carefully studies the features of paddy growth, and integrates the quantitative indicators of each growth stage as rice growth, thus providing a quantitative basis for rice growth prediction models.
2. The paper uses ElmanNN as the basic algorithm for rice growth prediction research. A rice growth prediction model based on ElmanNN was constructed. In the test, it was found that the ElmanNN is easy to fall into the local extreme value, which leads to a large deviation of individual points. After analyzing a variety of optimization methods, the genetic algorithm is finally accustomed to optimize the weight and threshold of the ElmanNN efficiency, reducing the possibility of trapping in local extrema. Simultaneously, the adaptive mechanism is introduced into the selection of the crossover operator and mutation operator of the algorithm, and the values of the crossover probability and mutation probability are dynamically adjusted, which not only ensures the diversity but also improves the search ability of the algorithm and finally makes the ameliorate rice growth prediction. Model accuracy has been ameliorating.

### 5.2. Prospect

The comparison experiment of the standard Elman network model verifies the prediction accuracy of the ameliorate model. On this basis, the prototype system of paddy upgrowth prediction is realized, and the specific functions of the acquisition layer, transmission layer, service layer, presentation layer, and other layers are introduced, and the task modules undertaken by them are emphasized, and the final prediction interface is displayed. In the specific field of paddy upgrowth prediction, when predecessors used neural networks to study paddy upgrowth, they did not go deep into multitudinous growth stages to deal with the effects of growth characteristics on yield in stages. The paper defines the concept of paddy upgrowth, builds a growth prediction model in stages, finally integrates yield prediction, and initially realizes the final research results, builds a prototype system for paddy upgrowth prediction, and realizes the growth of rice at different growth stages and prediction function. The constructed paddy upgrowth prediction model has basically achieved the expected results, but due to my limited ability and experimental conditions, this model still has several shortcomings that need to be ameliorated urgently. [25].

1. The sample data is further ameliorated. The sample data all come from one place, resulting in insufficient sample breadth and limited model applicability. The training samples will be further expanded in the later stage.
2. The dimension of circumstance element is further increased. Due to the limited experimental conditions, the selected environmental quantities may not be comprehensive and effective. At present, only a few environmental quantities that have a significant collision on yield are considered. However, under certain circumstances, there are relatively a larger part other circumstance element that cannot be ignored. These effects have not been fully taken into account.
3. The prototype system lacks the function of the intermediate protocol conversion layer. In the prototype system built on the basis of the model, the acquisition terminal may come from a designated manufacturer. In actual application scenarios, there are heterogeneous protocol systems such as multimanufacturers, and the protocols are not completely mutual and open. It is necessary to add a unified protocol conversion layer middleware to achieve unified access of the prototype system to each hardware.

## Figures and Tables

**Figure 1:** Flowchart of the improved Elman neural.

**Figure 2:** ElmanNN structure diagram.

**Table 1:** The number of hidden layer nodes and the total error in neural network simulation.

Quantity hidden layer nodes	Overall error	Quantity hidden layer nodes	Overall error
4	9.26e-04	5	4.24e-05
6	8.45e-05	7	9.31e-04
8	6.21e-04	9	2.45e-04
10	4.57e-04	11	3.56e-05
12	7.62e-05	13	2.73e-04

**Table 2:** Comparison of the errors of each algorithm.

Types of neural networks	Average mean square error	Average mean absolute error
BP neural network	0.00712	0.05423
ElmanNN	0.01045	0.08440
Ameliorate ElmanNN	0.00613	0.02603

## Data Availability

The dataset can be accessed upon request.
